This article has been retracted.

# Human Gut Microbiota: Dysbiosis and Manipulation

**DOI:** 10.3389/fcimb.2012.00123

**Published:** 2012-09-27

**Authors:** Dongqian Shen, Chuan Liu, Ran Xu, Faxing Zhang

**Affiliations:** ^1^Beijing Genomics Institute-ShenzhenShenzhen, China

The adult human intestine is home to an almost inconceivable number of microorganisms. Their population is up to 100 trillion, nearly 10 times larger than the total number of our somatic and germ cells. All three domains, including bacteria, archaea, and eukarya, are contained in the adult human gastrointestinal (GI) tract and the bacteria achieve the highest cell densities and phylogenetic diversities (Whitman et al., 1998). Such gut microbiome can be viewed as a microbial organ placed within a host organ and the genomes of our affiliated microbial partners (the microbiome) may contain more than 100 times the number of genes in our genome. Once established, the indigenous microbiota provides many crucial functions to the host endows us with functional features that we have not had to evolve ourselves (MacDonald and Monteleone, 2005). These have been reviewed elsewhere (Ley et al., 2009; Neish, 2009) and include the contribution to digestion (such as the ability of microbes to break down host non-digestible polysaccharides) and its secondary benefits (the generation of SCFA), the metabolism of xenobiotics, the development of human immune system, and the colonization resistance. Generally, a healthy human state is a homeostasis between the microbiota and the host. Maladies such as Crohn's disease, chronic periodontitis, and bacterial vaginosis are characterized by a disruption of this homeostasis, a state known as dysbiosis (Tamboli et al., 2004). Meanwhile, the composition of the intestinal microbiota can undergo dynamic changes as a result of its interactions with diet, genotype/epigenetic composition, and immune-metabolic function (Kau et al., 2011). We envision a future in which new therapeutics and diagnostics enable the management of our microbiota to treat and prevent disease. Here, the relationship between gut microbiome and diseases and the effort in adjusting the gut microbiome will be discussed briefly.

## The Human Gut Microbiota and Diseases

The human gut harbors diverse microbes that play a fundamental role in the health of their host. It differs from person to person depending on the unique species of bacteria accumulated over a lifetime. This means that every person's health is distinctly influenced by the specific byproducts created by their particular microbiota (Goodacre, 2007). Microbiome, considered as our “forgotten organ,” has been studied by some large-scale international projects such as HMP (Turnbaugh et al., 2007; Peterson et al., 2009) and MetaHIT (Qin et al., 2010). Based on an increasing number of studies on human microbiome, including the microbial community structure and function (Huttenhower et al., 2012), the researchers are shifting their concerns to the role of human microbiota in development of some acute or chronic diseases, especially GI Disorder. And the understanding that pathogenesis of some diseases is associated with result of complex interactions between microbiota and host was accepted more and more commonly.

The most frequently reported disease that has been proved to associate with dramatic changes in the gut microbiota is Inflammatory Bowel Disease (IBD; Dicksved et al., 2008). MacFarlane et al. (2009) revealed significant reductions in *Bifidobacterium* populations in rectal biopsies from IBD patients. Zhang et al. (2007) have shown that bacterial diversity of *Lactobacilli* varied greatly between ulcerated tissue and non-ulcerated tissue in the same UC individuals. The number of mucosal adherent bacteria, such as invasive *E. coli*, *Proteobacteria*, *Enterobacteriaceae* are increased in IBD patients’ gut (Nagalingam and Lynch, 2012). Despite the involvement of microorganisms in inflammatory processes, antibiotic therapy was unsuccessful in IBD. However, recent studies demonstrated the use of probiotics, prebiotics, and synbiotics suggested the potential for controlling these diseases through manipulation of the composition of the gut microbiota, and direct interactions with the gut immune system (MacFarlane et al., 2009).

Obesity and type 2 diabetes (T2D), the most prevalent metabolic diseases worldwide, are considered to be induced by impact of the microbiota on our metabolic health. Turnbaugh et al. (2009) observed that obesity is associated with phylum-level changes in the microbiota, reduced bacterial diversity, and altered representation of bacterial genes and metabolic pathways. The hypothesis is that the microbiota in obese individuals can harvest the more energy from food than the one in lean individuals. And another hypothesis is that gut microbiota can modulate plasma LPS levels which triggers chronic low-grade inflammation leading to obesity and diabetes (Cani et al., 2007). Another disease that related with obese tightly is non-alcoholic fatty liver. The intestinal microbiota may contribute to the development of non-alcoholic fatty liver disease through the complex and cooperative activities of two microbe-sensing protein families, namely nucleotide oligomerization domain receptors (NLRs) and Toll-like receptors (TLRs; Mukhopadhyay et al., 2011; Yeretssian, 2012), and through inflammasomes (Henao-Mejia et al., 2012) that shape metabolic pathway such as lipid accumulation.

The gut microbiota has a considerable impact on the host's intestinal immunity and immune responses. Rheumatoid Arthritis (RA), a systemic autoimmune disease, is considered to be linked with gut microbiome. The antibodies to *P. gingivalis* have been reported to be more frequent in RA subjects compared with controls and that the titer of RA-related autoantibodies and C-reactive protein concentrations are also higher in individuals infected with *P. gingivalis* suggesting that this organism plays a role in disease risk and progression in RA (Mikuls et al., 2009). Furthermore, RA is closely related to periodontal disease. In a case-control study, serum antibodies against disease-producing periodontal bacteria were identified more frequently in subjects affected by RA and periodontitis than control subjects (Ogrendik et al., 2005; Moen et al., 2006).

Commensal gut bacteria are essential to immune system development, and exposures disrupting the infant gut microbiota have been considered to be linked to asthma. The western diet has been found associated with increased risk of asthma for children (Nagel et al., 2010), and fast food consumption might counteract the protective effects of prolonged breastfeeding (Mai et al., 2009). Following birth, exclusive breastfeeding confers “beneficial” gut microbiota to infants, including increased colonization by *Bifidobacteria* and reduced prevalence and abundance of *C. difficile* compared to formula-fed infants (Penders et al., 2007; Fallani et al., 2010; Roger and McCartney, 2010). Infants who are not sufficiently exposed to *Bifidobacteria* in breast milk may have inappropriate immune responses to microbial exposures later in childhood, leading to atopic disorders including asthma. Beside of breast milk and other nutritional supplements, antibiotics affecting colonization of the intestinal bacteria by suppressing commensal bacteria, and causing the emergence of asthma-associated pathogens such as *C. difficile* are the next most commonly ingested substances by infants. The research shows that antibiotic use in the immediate period after birth can severely alter the composition and population of gut microbiota in infants (Fallani et al., 2010). Additional, the perinatal prevention from asthma via the intestinal microbiome is a relatively new perspective that has evolved long side modern technologies for the study of microbial communities (Azad and Kozyrskyj, 2012).

## The Pursue of Manipulate The Gut Microbiota

The increasingly serious chronic health issues, ranging from obesity and diabetes to bowel disease and RA, are being demonstrated to be linked with perturbations in gut flora. Hence, it is feasible to treat these complex diseases through adjusting the gut microbiome. Modern medicine is struggling to seek methods of treating these multi-component diseases. The ancient medical philosophies and practices of Asia – particularly those of traditional Chinese medicine (TCM) – can offer an alternative approach. TCM's reliance on complex mixtures of compounds and its philosophy – complete system needs to be balanced – of treating the human body, match up well with the synergistic properties of the gut microbiome (Crow, 2011). In addition, most herbal medicines are orally administered, which will result in the unavoidable exposure of these medicines to the microorganisms in the gut. During this process, some of them are selectively metabolized into active or absorbable components by enzymes derived from intestinal microbiota. Then the therapeutic effects can be achieved.

The Chinese microbiologist Zhao (2012) adopted a regimen involving Chinese yam and bitter melon – fermented prebiotic foods – that are believed to change the growth of bacteria in the digestive system. When he adopted the regimen by combing these prebiotics with diet composed of whole grains, he lost 20 kg in 2 years. Furthermore, his blood pressure, heart rate, and cholesterol level came down as well. The content of *Faecalibacterium prausnitzii*, a bacterium with anti-inflammatory properties, increased from an undetectable level to 14.5 percentage. of his total gut bacteria. The animal experiments showed that when rats were given a high fat diet (HFD) together with berberine, the major pharmacological component of the Chinese herb *Coptis chinensis* or Huanglian, they did not develop obesity or insulin resistance. What is more, the populations of known pathogens decreased while those of known beneficial bacteria increased in the gut. Other studies in mice also showed that the change from a low fat, plant polysaccharide diet to a western diet high in sugar, and fat would rapidly and profoundly reconfigure the composition of microbes in the gut. The gut microbiota in response to HFD feeding may allow the host to harvest more energy from food (Ley et al., 2005; Ley et al., 2006; Sanderson et al., 2006).

## Challenge and Prospect

Though the development of human gut microbiome research burst in the last decade, we are still unenlightened in facing to the complex gut composition and its influence on human health. Several challenges remain to be overcome in a near future. Firstly, the list of the diseases that related to the gut microbiome is just growing and growing, and these diseases are usually complex in terms of both pathogenesis and complication, while sequencing and computational technologies would be a bottleneck in large-scale correlation analysis between the human microbiome and diseases. Secondly, despite a growing number of researches discovered the relationship between alterations in the gut microbiome and diseases, it remains to be established whether these are causes or effects. Further studies are required to distinguish disease-associated changes from a mass of interindividual variations that observed in the microbiome. Thirdly, time-series studies of individuals to monitor the status alter process from health to disease and back to the health is necessary for exploring the changeable human microbiome. High-resolution time-series studies provide a feasibility to discriminate between “normal” perturbations and pathologic states, and between organisms that are simply passing through a body habitat and are entrenched residents of an ecosystem (Eckburg et al., 2005; Palmer et al., 2007; Koenig et al., 2011). In some studies, (Huse et al., 2008; Dethlefsen and Relman, 2010) rapid decreases in alpha diversity and a characteristic shift in community composition were observed in association with antibiotic therapy, followed by a rapid post-antibiotic increase in diversity as the gut community returned to a state similar (but not identical) to the pre-treatment state. Furthermore, despite a large number of reports have showed the different gut microbiome between patient and healthy person, the definition of “the healthy gut microbiome” remains unclear. And the methodologies that can change the unhealthy gut microbiome to a healthy one are still in investigation.

In terms of its application of human gut microbiome for human health development, we propose to monitor the microbiome when being healthy, and to establish a baseline indicating healthy, with more intensive monitoring when being sick and during treatment period. Such method demands the development of new diagnostic tools that are both accurate and sufficiently rapid to inform decisions regarding therapeutics. Such diagnostics are not yet feasible, but given recent advances in our ability to survey the human microbiome, this possibility is not far in the future, especially if we are able to identify particular components of the human microbiome that contribute disproportionately to the maintenance of human health. An adaptive management approach to clinical medicine provides a wonderful example of personalized medicine, with treatments tailored to individuals on the basis of diagnostic changes in an individual's microbiome, and continually adjusted through regular monitoring. Such an information-intensive approach, guided by ecological theory, has the potential to revolutionize the treatment of disease.
